The article "Gadolinium-Free Cardiac MR Stress T1-Mapping to Distinguish Epicardial From Microvascular Coronary Disease" was retracted in 2020. Reasons: fabricated or falsified data; fabricated or falsified images; an official misconduct investigation; misconduct by an author.

# Gadolinium-Free Cardiac MR Stress T1-Mapping to Distinguish Epicardial From Microvascular Coronary Disease

**DOI:** 10.1016/j.jacc.2017.11.071

**Published:** 2018-03-06

**Authors:** Alexander Liu, Rohan S. Wijesurendra, Joanna M. Liu, Andreas Greiser, Michael Jerosch-Herold, John C. Forfar, Keith M. Channon, Stefan K. Piechnik, Stefan Neubauer, Rajesh K. Kharbanda, Vanessa M. Ferreira

**Affiliations:** a Oxford Centre for Clinical Magnetic Resonance Research, Division of Cardiovascular Medicine, Radcliffe Department of Medicine, University of Oxford, Oxford, United Kingdom; b Siemens Healthcare GmbH, Erlangen, Germany; c Brigham and Women’s Hospital, Radiology, Cardiovascular Imaging, Boston, Massachusetts; d Oxford Heart Centre, John Radcliffe Hospital, Oxford, United Kingdom; e Division of Cardiovascular Medicine, Radcliffe Department of Medicine, University of Oxford, Oxford, United Kingdom

**Keywords:** adenosine stress, cardiac magnetic resonance, coronary artery disease, myocardial ischemia, T1 mapping, AUC, area under the receiver-operating characteristic curve, CAD, coronary artery disease, CI, confidence interval, CMD, coronary microvascular dysfunction, CMR, cardiac magnetic resonance, GBCA, gadolinium-based contrast agents, FFR, fractional flow reserve, IMR, index of microcirculatory resistance, LGE, late gadolinium enhancement, ROC, receiver-operating characteristic

## Abstract

**Background:**

Novel cardiac magnetic resonance (CMR) stress T1 mapping can detect ischemia and myocardial blood volume changes without contrast agents and may be a more comprehensive ischemia biomarker than myocardial blood flow.

**Objectives:**

This study describes the performance of the first prospective validation of stress T1 mapping against invasive coronary measurements for detecting obstructive epicardial coronary artery disease (CAD), defined by fractional flow reserve (FFR <0.8), and coronary microvascular dysfunction, defined by FFR ≥0.8 and the index of microcirculatory resistance (IMR ≥25 U), compared with first-pass perfusion imaging.

**Methods:**

Ninety subjects (60 patients with angina; 30 healthy control subjects) underwent CMR (1.5- and 3-T) to assess left ventricular function (cine), ischemia (adenosine stress/rest T1 mapping and perfusion), and infarction (late gadolinium enhancement). FFR and IMR were assessed ≤7 days post-CMR. Stress and rest images were analyzed blinded to other information.

**Results:**

Normal myocardial T1 reactivity (ΔT1) was 6.2 ± 0.4% (1.5-T) and 6.2 ± 1.3% (3-T). Ischemic viable myocardium downstream of obstructive CAD showed near-abolished T1 reactivity (ΔT1 = 0.7 ± 0.7%). Myocardium downstream of nonobstructive coronary arteries with microvascular dysfunction showed less-blunted T1 reactivity (ΔT1 = 3.0 ± 0.9%). Stress T1 mapping significantly outperformed gadolinium-based first-pass perfusion, including absolute quantification of myocardial blood flow, for detecting obstructive CAD (area under the receiver-operating characteristic curve: 0.97 ± 0.02 vs. 0.91 ± 0.03, respectively; p < 0.001). A ΔT1 of 1.5% accurately detected obstructive CAD (sensitivity: 93%; specificity: 95%; p < 0.001), whereas a less-blunted ΔT1 of 4.0% accurately detected microvascular dysfunction (area under the receiver-operating characteristic curve: 0.95 ± 0.03; sensitivity: 94%; specificity: 94%: p < 0.001).

The article "Gadolinium-Free Cardiac MR Stress T1-Mapping to Distinguish Epicardial From Microvascular Coronary Disease" was retracted in 2020. Reasons: fabricated or falsified data; fabricated or falsified images; an official misconduct investigation; misconduct by an author.

**Conclusions:**

CMR stress T1 mapping accurately detected and differentiated between obstructive epicardial CAD and microvascular dysfunction, without contrast agents or radiation.

In patients with angina, accurate diagnosis of myocardial ischemia is important for guiding clinical management (1). Invasive methods, such as fractional flow reserve (FFR) and the index of microcirculatory resistance (IMR), can assess the severity of epicardial coronary artery disease (CAD) and coronary microvascular dysfunction (CMD), respectively 2, 3, and are commonly evaluated during invasive angiography.

A novel cardiac magnetic resonance (CMR) technique, known as T1 mapping, has shown considerable promise for the noninvasive assessment of ischemia when performed during vasodilatory stress 4, 5. In magnetic resonance, T1 relaxation time is a magnetic property of tissue that prolongs with increased free water content 6, 7. T1 mapping displays the T1 values of imaged tissues on a pixel-by-pixel basis, enabling quantitative myocardial tissue characterization. Downstream of obstructive CAD, the microcirculation in ischemic myocardium undergoes compensatory vasodilation, which increases the myocardial blood volume 8, 9. This process increases the free water content in the ischemic myocardium, which is detectable by using T1 mapping 4, 5.

In a recent proof-of-concept study (4), we showed that adenosine stress and rest T1 mapping can distinguish between normal, ischemic, infarcted, and remote myocardium without the need for gadolinium contrast agents (Figure 1). Normal myocardium in control subjects exhibited normal resting T1, with significant positive T1 reactivity during adenosine vasodilatory stress (6.2 ± 0.5%). In patients with CAD, infarcted myocardium showed distinctively high resting T1, differentiating it from all other myocardial tissue classes, without significant T1 reactivity (0.2 ± 1.5%). Ischemic myocardium showed mildly (but significantly) elevated resting T1 compared with normal, without significant T1 reactivity (0.2 ± 0.8%). Remote (nonischemic/infarcted) myocardium in patients with CAD, although having normal resting T1, had a blunted T1 reactivity (3.9 ± 0.6%), possibly due to CMD. Normal, ischemic, infarcted, and remote myocardium have distinctive rest and stress T1 profiles that allow their differentiation from each other.

The article "Gadolinium-Free Cardiac MR Stress T1-Mapping to Distinguish Epicardial From Microvascular Coronary Disease" was retracted in 2020. Reasons: fabricated or falsified data; fabricated or falsified images; an official misconduct investigation; misconduct by an author.

**Figure 1:** Myocardial T1 at Rest and During Adenosine Stress at 1.5-T **(A)** T1 values at rest in normal and remote tissue were similar and significantly lower than in ischemic regions. Infarct T1 was the highest of all myocardial tissue but lower than the reference left ventricular blood pool of patients. During adenosine stress, normal and remote myocardial T1 increased significantly from baseline, whereas T1 in ischemic and infarcted regions remained relatively unchanged. **(B)** Relative T1 reactivity (δT1) in the patient’s remote myocardium was significantly blunted compared with normal and was completely abolished in ischemic and infarcted regions. All data indicate mean ± 1 SD. *p < 0.05.

Reprinted with permission from Liu et al. (4).

Based on these observations, we performed the first clinical validation of CMR stress T1 mapping against invasive coronary measures for detecting the following: 1) obstructive epicardial CAD, defined according to FFR <0.8; and 2) CMD, defined according to FFR ≥0.8 and IMR ≥25 U (10).

## Methods

### Study patients

We recruited 60 patients with stable angina and suspected CAD referred for outpatient diagnostic coronary angiography in a tertiary-referral hospital between February 2013 and December 2016. All 60 patients underwent CMR, followed within 7 days by invasive coronary angiography and physiology assessments. Healthy volunteers (n = 30) were also recruited to determine the normal ranges and interscan and intrascan variability of stress T1 mapping.

Exclusion criteria were unstable angina, New York Heart Association functional class IV heart failure, previous coronary artery bypass graft or valvular replacements, any valvular disease more than trivial in severity, and contraindications to magnetic resonance. The Oxford A Regional Ethics Committee, United Kingdom (Ref: 13/SC/0376), approved the study protocol. All participants provided written informed consent.

### Cardiac magnetic resonance

Patients underwent CMR at 2 commonly used clinical field-strengths: 1.5-T (n = 30; Magnetom Avanto; Siemens Healthcare GmbH, Erlangen, Germany) or 3-T (n = 30; Magnetom Trio, A Tim System; Siemens Healthcare GmbH) using established techniques as previously published (4). These included cine, adenosine stress and rest perfusion, and late gadolinium enhancement (LGE) imaging 4, 11.

The article "Gadolinium-Free Cardiac MR Stress T1-Mapping to Distinguish Epicardial From Microvascular Coronary Disease" was retracted in 2020. Reasons: fabricated or falsified data; fabricated or falsified images; an official misconduct investigation; misconduct by an author.

Adenosine stress and rest T1 mapping was performed before administration of any gadolinium-based contrast agents (GBCA), as previously described 4, 11. Briefly, native T1 maps were acquired first at rest by using the established, heart-rate independent Shortened Modified Look-Locker Inversion recovery T1 mapping technique (6) in 3 short-axis slice positions (basal, mid-ventricular, and apical) (4). Adenosine stress was given (140 to 210 μg/kg/min, 3 to 6 min, intravenously) before stress T1 maps were acquired in 3 short-axis slices matched to the resting T1 maps. Stress first-pass perfusion imaging was performed immediately after in matching slice positions to T1 maps, with an intravenous bolus of GBCA (0.03 mmol/kg at 6 ml/s; Dotarem; Guerbet, Villepinte, France) followed by a saline flush (15 ml at 6 ml/s). Matching rest perfusion images were acquired >15 min after stress perfusion and adenosine discontinuation. LGE imaging was performed in matching slice positions to cine and perfusion images 8 to 10 min after a top-up bolus of gadolinium (0.1 mmol/kg) (12).

Healthy control subjects underwent CMR at 1.5-T (n = 20) or 3-T (n = 10) using the same protocol as patients. To assess the interscan variability of stress myocardial T1 responses, 10 healthy volunteers who had CMR at 1.5-T had a repeat CMR >2 years later (mean: 3 ± 1 years) using the same protocol on the same scanner. To assess the intrascan variability of stress T1, in the repeat CMR scan, all 10 healthy volunteers underwent adenosine stress twice with a 15-min recovery period (Online Appendix).

All subjects (patients and control subjects) exhibited a significant hemodynamic response to adenosine stress (>10 beats/min increase in heart rate and ≥1 adenosine-related symptom [e.g., chest tightness]) (13). Furthermore, 60% of subjects also had a significant (>10 mm Hg) drop in systolic blood pressure.

### Invasive coronary physiology measurements

FFR and IMR were measured as previously described 2, 3, 10 by expert operators blinded to the research CMR results (Online Appendix). Significant epicardial coronary flow obstruction was defined by FFR <0.8 (3). Coronary microvascular dysfunction was defined by FFR ≥0.8 and IMR ≥25 U, where U denotes units or millimeter of mercury seconds 10, 14.

### Data analysis

T1 maps were analyzed as previously described 15, 16, by an experienced observer (A.L.) blinded to clinical information, invasive coronary data, and other CMR images. In brief, endocardial and epicardial borders were manually placed using dedicated in-house software MC-ROI (SKP in IDL, version 6.1, Exelis Visual Information Solutions, Boulder, Colorado), with care to avoid partial volume contaminations from surrounding tissues. CMR scans of healthy volunteers were analyzed in random order on a per-subject basis. For CMR scans of patients, T1 maps were segmented according to the American Heart Association’s 16-segment model (17), which generated a total of 1,920 myocardial segments (960 at rest and 960 during stress). To ensure maximal accuracy, only segments varying from good to excellent image quality were included, as previously described (15) (Online Appendix). Eight percent of myocardial segments were rejected in this quality control process, consistent with previous studies 15, 16, yielding 1,766 segments for final analysis. Separate analysis was also performed with inclusion of the rejected segments to assess the effect of this quality control process on final results.

The article "Gadolinium-Free Cardiac MR Stress T1-Mapping to Distinguish Epicardial From Microvascular Coronary Disease" was retracted in 2020. Reasons: fabricated or falsified data; fabricated or falsified images; an official misconduct investigation; misconduct by an author.

The mean segmental myocardial ΔT1 values were defined as: ([stress T1 − rest T1] / rest T1 × 100), and were allocated to each coronary territory according to the American Heart Association’s 16-segment model, accounting for coronary artery dominance, as previously described 4, 12, 16, 17. The segmental ΔT1 values were averaged to derive the mean ΔT1 for each coronary artery territory (17), which were then compared against the FFR and IMR, on a per-vessel basis.

Myocardial perfusion images were analyzed by using the 3 available techniques: visually (R.S.W. and A.L.), semi-quantitatively using myocardial perfusion reserve index (J.M.L.), and absolute quantification of myocardial blood flow to derive the myocardial perfusion reserve (J.M.L. and A.L.), as previously described 4, 18, 19, blinded to clinical information, T1 maps, and invasive coronary data (Online Appendix). Similar to T1 maps, myocardial perfusion images also underwent stringent quality control to ensure maximal accuracy of the data used for analysis; 7% of segment were rejected due to image artifacts (20), yielding 1,786 segments for final analysis. Left ventricular cines and LGE were analyzed as previously described (J.M.L.) (4), blinded to clinical information, other CMR images, and invasive coronary data.

### Statistical analysis

Normally distributed data were expressed as mean ± SD. Paired samples were assessed by using the paired Student's *t*-test, and unpaired samples were assessed by using the unpaired Student's *t*-test. The diagnostic performance of CMR stress ΔT1 for detecting epicardial CAD and microvascular dysfunction was assessed by using receiver-operating characteristic (ROC) curves, reporting sensitivity, specificity, accuracy, positive predictive values, and negative predictive values with 95% confidence intervals (CIs) where appropriate. The area under the ROC curve (AUC) was reported with ±1 SE (21). Pairwise comparisons of ROC curves were performed as previously described by DeLong et al. Categorical data were compared by using the Fisher exact test. Interscan and intrascan variability in healthy control subjects was assessed by using the Bland-Altman method, reporting error with 1 SD. The effect size for distinguishing between significantly obstructive (FFR <0.8) and nonobstructive (FFR ≥0.8) coronary arteries was estimated by using Cohen’s d (22). Because patients with 2- to 3-vessel CAD contributed >1 FFR and IMR value per-patient to the analysis, the intraclass correlation coefficient was calculated to determine the design effect and need to adjust for clustering, as previously described (23). The intraclass correlation coefficient was low for FFR (0.006; 95% CI: –0.15 to 0.22) and IMR (0.02; 95% CI: –0.12 to 0.21), demonstrating that the intracoronary measurements were not significantly correlated within individual patients. Each FFR and IMR value was treated independently for per-vessel analysis of the relationships with CMR parameters. To further account for clustering, p < 0.01 (0.05 / 3, two-tailed) was considered statistically significant (MedCalc version 12.7.8, MedCalc Software, Ostend, Belgium).

The article "Gadolinium-Free Cardiac MR Stress T1-Mapping to Distinguish Epicardial From Microvascular Coronary Disease" was retracted in 2020. Reasons: fabricated or falsified data; fabricated or falsified images; an official misconduct investigation; misconduct by an author.

## Results

### Subject characteristics

Subject characteristics are summarized in Tables 1 and 2. During coronary angiography, 40% of patients had single-vessel angiographic disease (≥50% stenosis according to visual assessment), 22% of patients had 2-vessel disease, 8% had 3-vessel disease, and 30% had no significant angiographic disease (<50% stenosis by visual assessment). FFR and IMR were assessed in 138 coronary arteries; the remaining 42 coronary arteries could not be assessed due to chronic total occlusions (n = 14) or operator discretion (n = 28 [angiographically nonobstructive vessels that were too tortuous, with slow flow, or were angiographically complex]).

**Table 1:** Subject Characteristics

	Patients (n = 60)	Control Subjects (n = 30)	p Value
Age, yrs	66 ± 10	51 ± 15	0.07
Male	42 (70)	21 (70)	0.91
Risk factors			
Hypertension	29 (48)	0 (0)	–
Diabetes mellitus	16 (27)	0 (0)	–
Hypercholesterolemia	21 (35)	0 (0)	–
Family history of ischemic heart disease	21 (35)	0 (0)	–
Ex-smoker	15 (25)	0 (0)	–
Medication			
Aspirin	50 (83)	0 (0)	–
ACE inhibitors/ARBs	24 (40)	0 (0)	–
Beta-blocker	54 (90)	0 (0)	–
Calcium-channel blocker	25 (42)	0 (0)	–
Clopidogrel	12 (20)	0 (0)	–
Nicorandil	8 (13)	0 (0)	–
Nitrate	4 (7)	0 (0)	–
Statin	38 (63)	0 (0)	–
Coronary angiography			
1-vessel CAD (≥50% stenosis)	24 (40)	–	–
2-vessel CAD	13 (22)	–	–
3-vessel CAD	5 (8)	–	–
3-vessel NOCAD (<50% stenosis)	18 (30)	–	–
Intracoronary (FFR and IMR) measurements			
No. of vessels assessed of the 180 available	138 (77)	–	–
Vessels with downstream myocardial infarction	13 (9)	–	–
Vessels with no downstream myocardial infarction	125 (91)	–	–
FFR <0.8 and IMR ≥25 U	25 (20)	–	–
FFR <0.8 and IMR <25 U	16 (13)	–	–
FFR ≥0.8 and IMR ≥25 U	35 (28)	–	–
FFR ≥0.8 and IMR <25 U	49 (39)	–	–

Values are mean ± SD or n (%).

The article "Gadolinium-Free Cardiac MR Stress T1-Mapping to Distinguish Epicardial From Microvascular Coronary Disease" was retracted in 2020. Reasons: fabricated or falsified data; fabricated or falsified images; an official misconduct investigation; misconduct by an author.

ACE = angiotensin-converting enzyme; ARB = angiotensin receptor blocker; CAD = coronary artery disease; FFR = fractional flow reserve; IMR = index of microcirculatory resistance; NOCAD = nonobstructive coronary artery disease.

**Table 2:** Cardiac Magnetic Resonance Data in Patients and Control Subjects

	Patients (n = 60)	Control Subjects (n = 30)	p Value
Age, yrs	66 ± 10	51 ± 15	0.07
Male	42 (70)	21 (70)	0.91
Cardiac magnetic resonance data			
Resting heart rate, beats/min	66 ± 9	66 ± 14	0.70
Stress heart rate, beats/min	91 ± 12	96 ± 13	0.51
Resting systolic blood pressure, mm Hg	142 ± 21	134 ± 16	0.13
Stress systolic blood pressure, mm Hg	131 ± 18	128 ± 18	0.45
Left ventricular ejection fraction, %	62 ± 11	66 ± 5	0.11
Late gadolinium enhancement	13	–	–
25%–50% transmural extent	5	–	–
>50% transmural extent	8	–	–

Values are mean ± SD, n (%), or n.

### Myocardial stress T1: Normal values and reproducibility

Healthy control subjects had normal resting T1, with normal T1 reactivity (ΔT1): 6.2 ± 0.4% (1.5-T) and 6.2 ± 1.3% (3-T) (Tables 3 and 4); T1 reactivity (ΔT1) was not significantly different between 1.5-T and 3-T. These findings are consistent with previously reported values 4, 24. Stress T1 mapping was highly reproducible, with low interscan (0.18 ± 0.36%) and intrascan (0.05 ± 0.36%) errors (Bland-Altman plots, Online Figure 1).

**Table 3:** Myocardial T1 Values in Healthy Control Subjects and Patients With CAD at 1.5-T

	Control Subjects (n = 20)	Patients With CAD (n = 30)				p Value
	Normal Myocardium	Obstructive CAD (FFR <0.8)	CMD (FFR ≥0.8, IMR ≥25 U)	No Significant CAD (FFR ≥0.8, IMR <25 U)	Myocardial Infarction	
No. of vessels and patients	–	23 vessels in 18/30 patients	18 vessels in 13/30 patients	22 vessels in 15/30 patients	6 vessels in 6/30 patients	–
Resting T1, ms	957 ± 22	977 ± 16∗	945 ± 21†	947 ± 18†	1,024 ± 28∗†‡§	<0.001
Stress T1, ms	1,015 ± 23	985 ± 16∗	972 ± 21∗	995 ± 18∗‡	1,028 ± 28∗†‡§	<0.001
ΔT1, %	6.2 ± 0.4	0.8 ± 0.8∗	2.9 ± 0.8∗†	5.1 ± 0.7†‡	0.9 ± 0.7∗‡§	<0.001
Resting MBF	1.1 ± 0.2	1.1 ± 0.3	1.0 ± 0.2	1.1 ± 0.3	1.2 ± 0.3	0.54
Stress MBF	3.0 ± 0.5	1.6 ± 0.5∗	1.6 ± 0.6∗	2.4 ± 0.6∗†‡	1.2 ± 0.4∗†‡§	<0.001
MPR	2.8 ± 0.5	1.5 ± 0.6∗	1.6 ± 0.6∗	2.4 ± 0.6∗†‡	1.0 ± 0.2∗†‡§	<0.001
MPRI	2.0 ± 0.3	1.3 ± 0.5∗	1.3 ± 0.5∗	1.8 ± 0.4∗†‡	1.0 ± 0.2∗†‡§	<0.001

Values are mean ± SD.

ΔT1 is (stress T1 – resting T1) ÷ resting T1 × 100. All T1 and ΔT1 values are mean ± 1 SD. All statistical analyses were performed by using an analysis of variance with Bonferroni post hoc corrections.

The article "Gadolinium-Free Cardiac MR Stress T1-Mapping to Distinguish Epicardial From Microvascular Coronary Disease" was retracted in 2020. Reasons: fabricated or falsified data; fabricated or falsified images; an official misconduct investigation; misconduct by an author.

CMD = coronary microvascular dysfunction; MBF = myocardial blood flow; MPR = myocardial perfusion reserve (stress MBF ÷ rest MBF); MPRI = myocardial perfusion reserve index; other abbreviations as in Table 1.

∗ p < 0.01 compared with normal control subjects.

† p < 0.01 compared with ischemic myocardium downstream obstructive CAD (FFR <0.8).

‡ p < 0.01 compared with CMD (FFR ≥0.8; IMR ≥25 U).

§ p < 0.01 compared with no significant CAD (FFR ≥0.8; IMR <25 U).

**Table 4:** Myocardial T1 Values in Healthy Control Subjects and Patients With CAD at 3-T

	Control Subjects (n = 10)	Patients With CAD (n = 30)				p Value
	Normal Myocardium	Obstructive CAD (FFR <0.8)	CMD (FFR ≥0.8, IMR ≥25 U)	No Significant CAD (FFR ≥0.8, IMR <25 U)	Myocardial Infarction	
No. of vessels and patients	–	18 vessels in 16/30 patients	17 vessels in 11/30 patients	27 vessels in 18/30 patients	7 vessels in 7/30 patients	–
Resting T1, ms	1,196 ± 23	1,239 ± 30∗	1,206 ± 30†	1,205 ± 27†	1,312 ± 37∗†‡§	<0.001
Stress T1, ms	1,263 ± 32	1,247 ± 32∗	1,243 ± 31∗	1,265 ± 29†‡	1,319 ± 40∗†‡§	<0.001
ΔT1, %	6.2 ± 1.3	0.7 ± 0.5∗	3.1 ± 1.1∗†	5.0 ± 1.0†‡	0.5 ± 0.3∗‡§	<0.001
Resting MBF	1.1 ± 0.2	1.1 ± 0.4	1.0 ± 0.2	1.0 ± 0.3	1.1 ± 0.3	0.61
Stress MBF	3.0 ± 0.3	1.5 ± 0.5∗	1.8 ± 0.7∗	2.6 ± 0.7∗†‡	1.1 ± 0.4∗†‡§	<0.001
MPR	2.8 ± 0.4	1.4 ± 0.5∗	1.8 ± 0.7∗	2.6 ± 0.7∗†‡	1.0 ± 0.3∗†‡§	<0.001
MPRI	2.0 ± 0.3	1.2 ± 0.3∗	1.2 ± 0.2∗	1.8 ± 0.5∗†‡	1.0 ± 0.3∗†‡§	<0.001

Values are mean ± SD.

ΔT1 is (stress T1 – resting T1) ÷ resting T1 × 100. All T1 and ΔT1 values are mean ± 1 SD. All statistical analyses were performed by using an analysis of variance with Bonferroni post hoc corrections.

Abbreviations as in Tables 1 and 3.

∗ p < 0.01 compared with normal control subjects.

† p < 0.01 compared with ischemic myocardium downstream of obstructive CAD (FFR <0.8).

‡ p < 0.01 compared with CMD (FFR ≥0.8; IMR ≥25 U).

§ p < 0.01 compared with no significant CAD (FFR ≥0.8; IMR <25 U).

### Stress T1 of infarcted myocardium

In patients, myocardial infarct scars (>25% transmural extent on LGE images) were present downstream of 9% (13 of 138) of coronary arteries (FFR: 0.8 ± 0.2). Infarcted segments had significantly elevated resting T1 values, with abolished stress myocardial T1 reactivity (ΔT1: 0.7 ± 0.7%) (Tables 3 and 4), similar to previous reports 4, 25. The remaining 91% (125 of 138) of coronary arteries had no downstream myocardial infarction.

### Myocardial stress T1 clearly distinguished between obstructive and nonobstructive coronary territories

Of the 125 viable coronary artery territories, 41 were downstream of obstructive (FFR <0.8) epicardial CAD, and 84 were downstream of nonobstructive (FFR ≥0.8) coronary arteries (3). On gadolinium first-pass perfusion CMR, myocardium downstream of obstructive CAD had significantly lower myocardial perfusion reserve compared with downstream of nonobstructive vessels (myocardial perfusion reserve: 1.4 ± 0.4 vs. 2.3 ± 0.6; p < 0.001) (23). On gadolinium-free CMR stress T1 mapping, myocardium downstream of obstructive CAD had significantly lower ΔT1 compared with downstream of nonobstructive vessels (ΔT1: 0.7 ± 0.7% vs. 4.1 ± 1.3%, respectively; p < 0.001), independent of magnetic field-strengths between 1.5- and 3-T. Tables 3 and 4 present breakdowns of CMR stress T1 and first-pass perfusion values according to FFR, IMR, and magnet field strength. There was a moderate correlation between percent stenosis severity and stress myocardial ΔT1 (rho = –0.46; p < 0.001) (Online Figure 2).

The article "Gadolinium-Free Cardiac MR Stress T1-Mapping to Distinguish Epicardial From Microvascular Coronary Disease" was retracted in 2020. Reasons: fabricated or falsified data; fabricated or falsified images; an official misconduct investigation; misconduct by an author.

The effect size for distinguishing between myocardium downstream of obstructive (FFR <0.8) CAD and nonobstructive (FFR ≥0.8) coronary arteries using CMR stress T1 mapping (Cohen’s d 3.3) was almost twice as large as for stress perfusion CMR (Cohen’s d 1.7). Figure 2 presents representative native T1 maps of a patient with CAD.

**Figure 2:** Noninvasive Assessment of Myocardial Ischemia Using Gadolinium-Free CMR Stress T1 Mapping A 69-year-old male patient presented with angina for 3 months. On angiography, he had 2 significant right coronary artery (RCA) stenoses **(black arrows)**, with a combined vessel fractional flow reserve (FFR) of 0.45, indicating coronary ischemia. The 1.5-T cardiac magnetic resonance (CMR) before coronary angiography showed an elevated resting T1 and reduced stress T1 response in the RCA territory (T1_rest_ 993 ms to T1_stress_ 999 ms: ΔT1 = 0.7%). Percutaneous coronary intervention (PCI) relieved the stenoses with good angiographic result **(white arrows)** and normalization of vessel FFR to 0.95. This finding was accompanied by significant improvements in the rest and stress T1 responses (T1_rest_ 956 ms to T1_stress_ 994 ms: ΔT1 = 4.0%).

### CMR stress ΔT1 had excellent diagnostic performance

A stress ΔT1 cutoff of 1.5% clearly distinguished between myocardium downstream of obstructive (FFR <0.8) and nonobstructive (FFR ≥0.8) coronary arteries (Figure 3). The blunted myocardial ΔT1 threshold of 1.5% showed excellent diagnostic performance for detecting functionally obstructive (FFR <0.8) epicardial CAD on ROC analysis (AUC: 0.97 ± 0.02; p < 0.001) (Figure 4), with a sensitivity of 93% (95% CI: 80% to 99%), specificity of 95% (95% CI: 88% to 99%), accuracy of 95% (95% CI: 85% to 99%), positive predictive value of 91% (95% CI: 77% to 97%), and negative predictive value of 96% (95% CI: 90% to 99%). After re-analysis with inclusion of rejected T1 map segments due to artifacts, the AUC remained the same: 0.97 ± 0.02 (p < 0.001).

The article "Gadolinium-Free Cardiac MR Stress T1-Mapping to Distinguish Epicardial From Microvascular Coronary Disease" was retracted in 2020. Reasons: fabricated or falsified data; fabricated or falsified images; an official misconduct investigation; misconduct by an author.

**Figure 3:** Relationship Between CMR Stress Myocardial ΔT1 and Invasive FFR A ΔT1 threshold of 1.5% optimally distinguished myocardial territories downstream of coronary arteries with FFR <0.8 and FFR ≥0.8 (data from 125 vessels in 60 patients). True positives: 38 vessels in 31 of 60 patients; true negatives: 80 vessels in 53 of 60 patients; false positives: 3 vessels in 3 of 60 patients; false negatives: 4 vessels in 4 of 60 patients. Abbreviations as in Figure 2.

**Figure 4:** Diagnostic Performance of CMR Stress T1 Mapping (ΔT1) and Gadolinium Contrast–Enhanced Stress Perfusion for Detecting Obstructive CAD True positive: myocardial segments downstream of obstructive coronary arteries (FFR <0.8); true negative: myocardial segments downstream of nonobstructive coronary arteries (FFR ≥0.8). Area under the curve (AUC), all p < 0.001. Stress T1 mapping (AUC: 0.97 ± 0.02; p < 0.001) had significantly higher diagnostic performance than stress perfusion CMR by visual (AUC: 0.85 ± 0.04; p < 0.001), semi-quantitative (AUC: 0.87 ± 0.04; p < 0.001) and quantitative (AUC: 0.91 ± 0.03; p < 0.001) analyses for detecting obstructive FFR <0.8 epicardial coronary artery disease (CAD) (all comparisons p < 0.01). The different methods of perfusion CMR analysis did not differ significantly in diagnostic performance for detecting significant CAD (all p > 0.22). Data are based on 125 coronary artery territories in 60 patients. AUC = area under the receiver-operating characteristic curve; other abbreviations as in Figure 2.

CMR stress ΔT1 (AUC: 0.97 ± 0.02; p < 0.001) significantly outperformed stress gadolinium-based perfusion by visual (AUC: 0.85 ± 0.04; p < 0.001), semi-quantitative (AUC: 0.87 ± 0.04; p < 0.001), and quantitative (AUC: 0.91 ± 0.03; p < 0.001) analyses for detecting obstructive (FFR <0.8) epicardial CAD (all comparisons p < 0.01) (Figure 4). The diagnostic performance of gadolinium-based perfusion CMR was similar among the 3 methods of analysis (all p > 0.22). Re-analysis with inclusion of rejected perfusion segments (7%) did not significantly alter the diagnostic performance of visual (AUC: 0.85 ± 0.04; p < 0.001), semi-quantitative (AUC: 0.86 ± 0.04; p < 0.001), and quantitative (AUC: 0.90 ± 0.03; p < 0.001) analyses for detecting obstructive epicardial CAD (all p > 0.8).

### CMR stress ΔT1 can detect CMD

Downstream of obstructive (FFR <0.8) CAD, myocardium with IMR ≥25 U (10) had similar stress ΔT1 compared with myocardium with IMR <25 U (0.8 ± 0.6% vs. 0.7 ± 0.7%; p = 0.97), suggesting that the reduced coronary vasodilatory reserve in this setting is predominantly driven by epicardial coronary flow limitation.

The article "Gadolinium-Free Cardiac MR Stress T1-Mapping to Distinguish Epicardial From Microvascular Coronary Disease" was retracted in 2020. Reasons: fabricated or falsified data; fabricated or falsified images; an official misconduct investigation; misconduct by an author.

In contrast, downstream of nonobstructive (FFR ≥0.8) coronary arteries, myocardium with IMR ≥25 U demonstrated an impaired ΔT1 compared with myocardium with IMR <25 U (3.0 ± 0.9% vs. 5.0 ± 0.9%; p < 0.001). Importantly, this impaired myocardial ΔT1 of CMD (FFR ≥0.8 and IMR ≥25 U) was still significantly higher than the abolished myocardial ΔT1 downstream of obstructive epicardial CAD (3.0 ± 0.9% vs. 0.7 ± 0.7%; p < 0.001), which enabled distinction between these 2 pathological entities.

Downstream of nonobstructive (FFR ≥0.8) coronary arteries with IMR <25 U, the myocardial ΔT1 was similar to normal control subjects (5.0 ± 0.9% vs. 6.2 ± 0.8%; p = 0.17), suggesting the absence of significant epicardial or microvascular CAD. Characteristic patterns of stress and rest T1 values are shown in Tables 3 and 4.

Downstream of nonobstructive (FFR ≥0.8) coronary arteries, a ΔT1 threshold of 4.0% accurately detected coronary microvascular dysfunction (IMR ≥25 U) on ROC analysis (AUC: 0.95 ± 0.03; p < 0.001), with a sensitivity of 94% (95% CI: 81% to 99%), specificity of 94% (95% CI: 83% to 99%), accuracy of 94% (95% CI: 80% to 99%), positive predictive value of 92% (95% CI: 77% to 98%), and negative predictive value of 96% (95% CI: 86% to 100%). Furthermore, this ΔT1 threshold of 4.0% had similarly high diagnostic performance for detecting CMD in patients with all 3 nonobstructive vessels (18 patients, 50% male; AUC: 0.94 ± 0.03; p < 0.001) compared with patients who also have significant 1 or 2 obstructive epicardial CAD (30 patients, 70% male; AUC: 0.96 ± 0.03; p < 0.001). The diagnostic performance of stress T1 mapping and perfusion CMR to distinguish between obstructive epicardial CAD (FFR <0.8) and CMD (FFR ≥0.8 and IMR ≥25 U) are shown in Online Figure 3.

## Discussion

This study is the first to report the excellent diagnostic performance of CMR stress T1 mapping for detecting obstructive epicardial CAD, as defined by the clinical invasive reference standard (FFR <0.8) method. Stress T1 mapping significantly outperformed the current CMR standard for detecting obstructive CAD with stress gadolinium-based first-pass perfusion imaging, whether using visual, semi-quantitative, or quantitative analysis. Furthermore, stress T1 mapping accurately detected coronary microvascular dysfunction defined invasively by a high IMR value (≥25 U) downstream of nonobstructive (FFR >0.8) coronary arteries. This new noninvasive CMR biomarker offers the unique potential to detect and differentiate between epicardial obstructive CAD and coronary microvascular dysfunction (Central Illustration), with excellent interscan and intrascan reproducibility.

The article "Gadolinium-Free Cardiac MR Stress T1-Mapping to Distinguish Epicardial From Microvascular Coronary Disease" was retracted in 2020. Reasons: fabricated or falsified data; fabricated or falsified images; an official misconduct investigation; misconduct by an author.

**Central Illustration:** CMR Stress T1 Mapping for the Assessment of Epicardial and Microvascular CAD Assessment of epicardial coronary artery disease (CAD) and microvascular dysfunction using gadolinium-free cardiac magnetic resonance (CMR) stress T1-mapping (ΔT1). Each **dot** represents a noninfarcted coronary artery territory, totaling 125 territories in 60 patients. Obstructive epicardial CAD: 41 vessels in 34 of 60 patients; microvascular dysfunction: 35 vessels in 24 of 60 patients; nonobstructive coronaries: 49 vessels in 33 of 60 patients. Significant obstructive epicardial CAD was defined as fractional flow reserve (FFR) <0.8. Microvascular dysfunction was defined as FFR ≥0.8 and index of microcirculatory resistance (IMR) ≥25 U.

### CMR stress T1 mapping: Accurate assessment of obstructive epicardial CAD

CMR is well established in clinical guidelines as a multiparametric imaging modality for assessing patients with angina (1). In this study, CMR stress T1 mapping significantly outperformed stress perfusion imaging for detecting obstructive epicardial CAD. This finding indicates that the assessment of myocardial blood volume by stress T1 mapping may be a superior surrogate of ischemia than the assessment of myocardial blood flow by perfusion imaging. Myocardial blood volume is a sensitive marker of vasodilatory reserve downstream of obstructive CAD 8, 9, 26, 27, 28. Studies using contrast-enhanced echocardiography and CMR to estimate myocardial blood volume have shown that it is also related to alterations in myocardial oxygen consumption downstream of obstructive CAD 26, 29, 30. Furthermore, blood-oxygen-level-dependent imaging was recently used to assess myocardial oxygenation as a more direct marker of ischemia 31, 32. In addition to myocardial blood volume changes, the stress Shortened Modified Look-Locker Inversion recovery–T1 responses are likely to be enhanced by sensitivity to the underlying blood-oxygen-level-dependent effect (5) and possible arterial spin labeling effects (33). Therefore, stress T1 mapping reflects a wide range of effects related to vascular reactivity, with high diagnostic value for detecting significant CAD.

Downstream of obstructive CAD, significant microcirculatory vasodilation occurs, which maintains adequate myocardial perfusion with little change in resting myocardial blood flow (34). However, this compensatory vasodilation downstream of significant CAD causes an expansion of the myocardial intravascular space and an increase in myocardial blood volume 8, 9, 30. Hence, although myocardial blood flow at rest, as assessed quantitatively according to perfusion CMR, was similar downstream of obstructive and nonobstructive coronary arteries, there was a significant observed difference in resting myocardial T1. These likely different mechanisms for ischemia detection between CMR stress T1 mapping and stress perfusion could contribute to the differences in diagnostic performances in this study.

The article "Gadolinium-Free Cardiac MR Stress T1-Mapping to Distinguish Epicardial From Microvascular Coronary Disease" was retracted in 2020. Reasons: fabricated or falsified data; fabricated or falsified images; an official misconduct investigation; misconduct by an author.

As a novel diagnostic method, the stress myocardial ΔT1 values are characterized by tight reference ranges, with extremely low interscan and intrascan variability. Consequently, stress T1 mapping commanded a higher effect size than stress perfusion for differentiating between obstructive and nonobstructive CAD, despite an apparently modest range of change between 0% and approximately 6%. The results of this study set the stage for testing the wider diagnostic value of stress T1 mapping in a larger, multicenter study comprising an unselected patient population.

### CMR stress T1 mapping: Ischemia testing without contrast agents

Another advantage of CMR stress T1 mapping over stress perfusion imaging is the complete avoidance of GBCA administration. This approach circumvents any potential safety concerns regarding GBCA-related nephrogenic systemic fibrosis in patients with advanced renal failure (35), GBCA accumulation in the brain with repeat CMR scans (36), or allergic reactions to GBCA (37). Stress T1 mapping can potentially open the door for patients with advanced renal failure to benefit from accurate CMR-based ischemia assessment; this topic is an area of active research.

### CMR stress T1 mapping: Accurate assessment of CMD

More than one-half of patients with angina have nonobstructive coronary arteries on invasive angiography (38). Although these patients with “microvascular angina” are often reassured as having no significant CAD or are treated empirically with antianginal medication, they experience reduced quality of life and adverse long-term prognosis (39). Therefore, a noninvasive test to accurately detect CMD can improve clinical risk stratification and guide targeted therapy in patients with microvascular angina.

Stress T1 mapping may represent a breakthrough in this respect with the ability to noninvasively diagnose and differentiate between epicardial CAD and CMD. Myocardial territories downstream of obstructive epicardial (FFR <0.8) CAD had elevated resting T1, which augmented minimally with adenosine stress, leading to a near-zero stress T1 response. In contrast, myocardial territories downstream of nonobstructive coronary arteries had normal resting T1, and the presence of CMD (FFR ≥0.8 and IMR ≥25 U) is associated with a blunted and detectable stress T1 response compared with normal. Importantly, this blunted stress T1 reactivity in myocardium with CMD was less severe compared with myocardium downstream of obstructive epicardial CAD, which allows noninvasive differentiation between these 2 pathological conditions (Table 3). The distinctive diagnostic thresholds for obstructive epicardial CAD (ΔT1 <1.5%), CMD (ΔT1 1.5% to 4.0%), and normal (ΔT1 >4.0%) (Central Illustration) deserves further validation in a larger study with an unselected patient population.

The article "Gadolinium-Free Cardiac MR Stress T1-Mapping to Distinguish Epicardial From Microvascular Coronary Disease" was retracted in 2020. Reasons: fabricated or falsified data; fabricated or falsified images; an official misconduct investigation; misconduct by an author.

### Study limitations and future directions

This study examined the diagnostic performance of CMR stress T1 mapping for the detection of ischemia in native coronary arteries. The utility of stress T1 mapping for the detection of ischemia in more complex CAD, such as chronic total occlusion and after coronary artery bypass grafting, requires further investigation. A proportion of T1 map and stress perfusion segments (7% to 8%) was rejected in a stringent quality control process to ensure maximal accuracy in this validation study. Reassuringly, re-inclusion of these segments did not significantly affect the diagnostic performance of either method for detecting obstructive CAD. In this study, which focused on the detection of ischemia, the infarct scars were assessed by using LGE imaging. Although viable ischemic myocardium and infarcted myocardium both showed a near-zero stress T1 response, infarcted myocardium had significantly higher resting T1, which allowed differentiation from noninfarcted tissue without the need for LGE (4). This outcome requires further validation to develop a completely gadolinium-free protocol for assessing patients with CAD. Finally, this study paves the way for a larger multicenter study to determine the wider diagnostic value of stress T1 mapping in an all-comers population to guide clinical decision-making and predict long-term prognosis.

## Conclusions

CMR stress T1 mapping accurately detected and differentiated between obstructive epicardial CAD and CMD, without contrast agents or radiation.

Perspectives **COMPETENCY IN PATIENT CARE AND PROCEDURAL SKILLS:** In patients with angina, adenosine stress T1 mapping CMR can accurately distinguish obstructive epicardial CAD from CMD without exposure to radiation or gadolinium-based contrast.

**TRANSLATIONAL OUTLOOK:** Further research is required to clarify the clinical utility and prognostic value of this test in unselected patient populations.

## References

[1] Fihn S.D., Blankenship J.C., Alexander K.P. (2014). 2014 ACC/AHA/AATS/PCNA/SCAI/STS focused update of the guideline for the diagnosis and management of patients with stable ischemic heart disease: a report of the American College of Cardiology/American Heart Association Task Force on Practice Guidelines, and the American Association for Thoracic Surgery, Preventive Cardiovascular Nurses Association, Society for Cardiovascular Angiography and Interventions, and Society of Thoracic Surgeons. J Am Coll Cardiol.

The article "Gadolinium-Free Cardiac MR Stress T1-Mapping to Distinguish Epicardial From Microvascular Coronary Disease" was retracted in 2020. Reasons: fabricated or falsified data; fabricated or falsified images; an official misconduct investigation; misconduct by an author.

[2] Lee J.M., Jung J.H., Hwang D. (2016). Coronary flow reserve and microcirculatory resistance in patients with intermediate coronary stenosis. J Am Coll Cardiol.

[3] De Bruyne B., Fearon W.F., Pijls N.H. (2014). Fractional flow reserve-guided PCI for stable coronary artery disease. N Engl J Med.

[4] Liu A., Wijesurendra R.S., Francis J.M. (2016). Adenosine stress and rest T1 mapping can differentiate between ischemic, infarcted, remote, and normal myocardium without the need for gadolinium contrast agents. J Am Coll Cardiol Img.

[5] Piechnik S.K., Neubauer S., Ferreira V.M. (2017 Sep 15). State-of-the-art review: stress T1 mapping-technical considerations, pitfalls and emerging clinical applications. MAGMA.

[6] Piechnik S.K., Ferreira V.M., Dall'Armellina E. (2010). Shortened Modified Look-Locker Inversion recovery (ShMOLLI) for clinical myocardial T1-mapping at 1.5 and 3 T within a 9 heartbeat breathhold. J Cardiovasc Magnetic Resonance.

[7] Liu J.M., Liu A., Leal J. (2017). Measurement of myocardial native T1 in cardiovascular diseases and norm in 1291 subjects. J Cardiovasc Magnetic Resonance.

[8] Le D.E., Jayaweera A.R., Wei K., Coggins M.P., Lindner J.R., Kaul S. (2004). Changes in myocardial blood volume over a wide range of coronary driving pressures: role of capillaries beyond the autoregulatory range. Heart.

[9] Lindner J.R., Skyba D.M., Goodman N.C., Jayaweera A.R., Kaul S. (1997). Changes in myocardial blood volume with graded coronary stenosis. Am J Physiol.

[10] Lee B.K., Lim H.S., Fearon W.F. (2015). Invasive evaluation of patients with angina in the absence of obstructive coronary artery disease. Circulation.

[11] Liu A., Wijesurendra R.S., Ariga R. (2017). Splenic T1-mapping: a novel quantitative method for assessing adenosine stress adequacy for cardiovascular magnetic resonance. J Cardiovasc Magnetic Resonance.

[12] Ferreira V.M., Marcelino M., Piechnik S.K. (2016). Pheochromocytoma is characterized by catecholamine-mediated myocarditis, focal and diffuse myocardial fibrosis, and myocardial dysfunction. J Am Coll Cardiol.

[13] Kramer C.M., Barkhausen J., Flamm S.D., Kim R.J., Nagel E. (2013). Society for Cardiovascular Magnetic Resonance Board of Trustees Task Force on Standardized Protocols. Standardized cardiovascular magnetic resonance (CMR) protocols 2013 update. J Cardiovasc Magnetic Resonance.

The article "Gadolinium-Free Cardiac MR Stress T1-Mapping to Distinguish Epicardial From Microvascular Coronary Disease" was retracted in 2020. Reasons: fabricated or falsified data; fabricated or falsified images; an official misconduct investigation; misconduct by an author.

[14] Fearon W.F., Balsam L.B., Farouque H.M. (2003). Novel index for invasively assessing the coronary microcirculation. Circulation.

[15] Ferreira V.M., Piechnik S.K., Dall'Armellina E. (2012). Non-contrast T1-mapping detects acute myocardial edema with high diagnostic accuracy: a comparison to T2-weighted cardiovascular magnetic resonance. J Cardiovasc Magnetic Resonance.

[16] Ferreira V.M., Piechnik S.K., Dall'armellina E. (2013). T1 mapping for the diagnosis of acute myocarditis using CMR: comparison to T2-weighted and late gadolinium enhanced imaging. J Am Coll Cardiol Img.

[17] Cerqueira M.D., Weissman N.J., Dilsizian V. (2002). Standardized myocardial segmentation and nomenclature for tomographic imaging of the heart. A statement for healthcare professionals from the Cardiac Imaging Committee of the Council on Clinical Cardiology of the American Heart Association. Circulation.

[18] Cheng A.S., Pegg T.J., Karamitsos T.D. (2007). Cardiovascular magnetic resonance perfusion imaging at 3-Tesla for the detection of coronary artery disease: a comparison with 1.5-Tesla. J Am Coll Cardiol.

[19] Jerosch-Herold M., Swingen C., Seethamraju R.T. (2002). Myocardial blood flow quantification with MRI by model-independent deconvolution. Med Phys.

[20] Ferreira P.F., Gatehouse P.D., Mohiaddin R.H., Firmin D.N. (2013). Cardiovascular magnetic resonance artefacts. J Cardiovasc Magn Reson.

[21] DeLong E.R., DeLong D.M., Clarke-Pearson D.L. (1988). Comparing the areas under two or more correlated receiver operating characteristic curves: a nonparametric approach. Biometrics.

[22] Cohen J. (1988). Statistical Power Analysis for the Behavioral Sciences (2nd Edition).

[23] Lockie T., Ishida M., Perera D. (2011). High-resolution magnetic resonance myocardial perfusion imaging at 3.0-Tesla to detect hemodynamically significant coronary stenoses as determined by fractional flow reserve. J Am Coll Cardiol.

[24] Mahmod M., Piechnik S.K., Levelt E. (2014). Adenosine stress native T1 mapping in severe aortic stenosis: evidence for a role of the intravascular compartment on myocardial T1 values. J Cardiovasc Magnetic Resonance.

[25] Kuijpers D., Prakken N.H., Vliegenthart R. (2016). Caffeine intake inverts the effect of adenosine on myocardial perfusion during stress as measured by T1 mapping. Int J Cardiovasc Imaging.

[26] McCommis K.S., Goldstein T.A., Abendschein D.R. (2010). Roles of myocardial blood volume and flow in coronary artery disease: an experimental MRI study at rest and during hyperemia. Eur Radiol.

The article "Gadolinium-Free Cardiac MR Stress T1-Mapping to Distinguish Epicardial From Microvascular Coronary Disease" was retracted in 2020. Reasons: fabricated or falsified data; fabricated or falsified images; an official misconduct investigation; misconduct by an author.

[27] McCommis K.S., Goldstein T.A., Zhang H., Misselwitz B., Gropler R.J., Zheng J. (2007). Quantification of myocardial blood volume during dipyridamole and dobutamine stress: a perfusion CMR study. J Cardiovasc Magnetic Resonance.

[28] Moir S., Haluska B.A., Jenkins C., McNab D., Marwick T.H. (2005). Myocardial blood volume and perfusion reserve responses to combined dipyridamole and exercise stress: a quantitative approach to contrast stress echocardiography. J Am Soc Echocardiogr.

[29] Firschke C., Andrassy P., Linka A.Z., Busch R., Martinoff S. (2007). Adenosine myocardial contrast echo in intermediate severity coronary stenoses: a prospective two-center study. Int J Cardiovasc Imaging.

[30] McCommis K.S., Zhang H., Goldstein T.A. (2009). Myocardial blood volume is associated with myocardial oxygen consumption: an experimental study with cardiac magnetic resonance in a canine model. J Am Coll Cardiol Img.

[31] Arnold J.R., Karamitsos T.D., Bhamra-Ariza P. (2012). Myocardial oxygenation in coronary artery disease: insights from blood oxygen level-dependent magnetic resonance imaging at 3 Tesla. J Am Coll Cardiol.

[32] Friedrich M.G., Karamitsos T.D. (2013). Oxygenation-sensitive cardiovascular magnetic resonance. J Cardiovasc Magnetic Resonance.

[33] Wacker C.M., Fidler F., Dueren C. (2003). Quantitative assessment of myocardial perfusion with a spin-labeling technique: preliminary results in patients with coronary artery disease. J Magn Reson Imaging.

[34] Salerno M., Beller G.A. (2009). Noninvasive assessment of myocardial perfusion. Circ Cardiovasc Imaging.

[35] Bennett C.L., Qureshi Z.P., Sartor A.O. (2012). Gadolinium-induced nephrogenic systemic fibrosis: the rise and fall of an iatrogenic disease. Clinical Kidney J.

[36] McDonald R.J., McDonald J.S., Kallmes D.F. (2015). Intracranial gadolinium deposition after contrast-enhanced MR imaging. Radiology.

[37] Bruder O., Wagner A., Lombardi M. (2013). European Cardiovascular Magnetic Resonance (EuroCMR) registry—multinational results from 57 centers in 15 countries. J Cardiovasc Magnetic Resonance.

[38] Patel M.R., Peterson E.D., Dai D. (2010). Low diagnostic yield of elective coronary angiography. N Engl J Med.

[39] Jespersen L., Hvelplund A., Abildstrom S.Z. (2012). Stable angina pectoris with no obstructive coronary artery disease is associated with increased risks of major adverse cardiovascular events. Eur Heart J.

